# Influence of Lacidophilin Vaginal Capsules plus rh-IFN-*α*2b on Efficacy, Vaginal Microecology, and Safety of Patients with HPV Infection

**DOI:** 10.1155/2022/3632053

**Published:** 2022-08-03

**Authors:** Yan Sun, Jianqun Xu, Hongya Zhou, Lina You, Yan Zhu

**Affiliations:** Obstetrics and Gynecology, Xishan People's Hospital of Wuxi City, Wuxi 214000, Jiangsu, China

## Abstract

**Background:**

Human papillomavirus (HPV) is a self-limiting disease, and there is no specific antiviral drug at present.

**Purpose:**

Here, we analyzed the influence of lacidophilin vaginal capsules plus recombinant human interferon *α*-2b (rh-IFN-*α*2b) on efficacy, vaginal microecology, and safety of patients with HPV infection. Two hundred cases of HPV infection admitted between January 2019 and December 2020 were retrospectively collected. Of them, 90 cases receiving rh-IFN-*α*2b intervention were assigned to the control group (CG), and 110 cases given lacidophilin vaginal capsules in addition to rh-IFN-*α*2b were included in the research group (RG). Baseline data, efficacy, vaginal microecology, microecological restoration recovery, and incidence of adverse events (AEs) were compared between the two groups.

**Results:**

The analyses revealed nonsignificant difference in baseline data between RG and CG, indicating comparability. In terms of efficacy, RG showed a statistically higher negative conversion ratio (NCR) than CG (57.27% vs. 47.78%), as well as an obviously higher overall response rate (ORR) (90.90% vs. 72.22%). As far as the vaginal microecology was concerned, the incidence rates of catalase-positive, sialidase-positive, abnormal microbial density, and abnormal microbial diversity of RG were significantly lower compared with CG, but no evident differences were determined in *Trichomonas vaginalis*-positive and *Candida*-positive. As for microecological restoration, RG had an obviously higher vaginal microecological recovery rate than CG (90.00% vs. 65.56%), as well as notably lower vaginal secretion pH and Nugent score. On the other hand, RG and CG showed no statistical significance in the incidence of AEs (12.73% vs. 13.33%).

**Conclusions:**

The main contributions of this study are as follows: first, it is confirmed that lacidophilin vaginal capsules plus rh-IFN-*α*2b has better clinical effects than rh-IFN-*α*2b alone in HPV-infected patients; second, it demonstrates that the combination therapy can significantly improve NCR and ORR, without increasing the incidence of AEs, and is beneficial to improve patients' vaginal microecology and promote its restoration from the multidimensional aspects of efficacy, safety, and vaginal microecology and its recovery. Our findings provide valuable clinical evidence for the drug treatment of HPV-infected patients.

## 1. Introduction

Human papillomavirus (HPV) infection is highly correlated with cervical cancer (CC, including squamous intraepithelial lesion (SIL)), in which persistent high-risk HPV can cause at least 90% of CC cases and is closely associated with squamous intraepithelial lesions [1, 2]. As a carcinogenic factor, HPV infection can also cause cancers in the vulva, anus, and oropharynx [3]. The carcinogenic mechanism of HPV infection is shown to be related to vaginal microecology, inflammatory factors, genetics, and immune function [4, 5]. This study analyses the clinical effect of drug therapy on HPV infection, aiming to provide novel references for the improvement of vaginal microecology and alleviation of inflammatory factors in HPV-infected patients.

Interferon *α*-2b is essentially a cytokine protein that is widely used in virtue of its broad-spectrum antitumor, antivirus, and immune-enhancing effects [6]. With the same biological function, recombinant human interferon *α*-2b (rh-IFN-*α*2b) can exert antitumor action in combination with other drugs [7]. In the research of Kaliki et al. [8], it is pointed out that rh-IFN-*α*2b can be used to treat ocular surface squamous tumor, which is a cost-effective alternative to surgery and can play an immunotherapy role in this disease. Song et al. [9] reported that interferon *α*-2b can be combined with paclitaxel and 13-cis-retinoic acid to act on advanced and recurrent CC, with satisfactory efficacy and safety. Another drug, lacidophilin vaginal capsule is a living bacterium preparation based on lactic acid bacteria (LAB), which can not only improve vaginal microecological flora and abnormalities of acid-base balance but also has a reactivation effect on vaginal immune defense [10]. It is worth mentioning that HPV infection will lead to the imbalance of vaginal microecology, disrupting the checks, and balances between LAB and other microorganisms [11]. Given the current lack of research on the application of lacidophilin vaginal capsules plus rh-IFN-*α*2b in treating HPV-infected patients, we conduct relevant research in the hope of providing novel insights into the treatment of patients with HPV infection.

## 2. Data and Methods

### 2.1. Study Population

Inclusion criteria were as follows: diagnosis of HPV single infection or low-grade squamous intraepithelial lesion (LSIL); treatment-naive patients; nonpregnancy and nonlactating women; normal cognitive and mental conditions; premenopausal women; high compliance; and no contraindications to the medication used in this study.

Exclusion criteria were as follows: malignant tumors; one or more organ dysfunction; abnormalities of immune, hematopoietic or coagulation functions; distant metastasis; and presence of acute phase gynecological inflammation.

After rigorous screening, 200 HPV-infected patients admitted between January 2019 and December 2020 were enrolled, including 90 cases (control group, CG) treated with rh-IFN-*α*2b and 110 cases (research group, RG) additionally given lacidophilin vaginal capsules. The mean age and average course of disease of CG were 29.71 ± 5.68 years and 2.25 ± 1.05 years, respectively, while in RG, the data were 30.76 ± 8.14 years, and 2.49 ± 1.19 years, respectively. All subjects provided informed consent, and this study has been ethically ratified by our hospital.

### 2.2. Therapeutic Methods

CG received rh-IFN-*α*2b intervention. The subjects washed the vulva every night before going to bed since the third day after menstruation and placed the drug deep (one pill/time) in the vagina to the fornix near the cervical orifice once every two days. With ten times as a course of treatment, the patients were treated for a total of three courses.

RG was additionally intervened by the drug lacidophilin vaginal capsules, which was administered the second night after the use of rh-IFN-*α*2b intervention, two capsules at a time, using the same method as mentioned above. The patients received 4 courses of treatment, with seven times of medication as a course.

Antibiotics, vaginal irrigation, tub bath, and sexual life were prohibited in both the groups during treatment. Efficacy assessment was performed three months after treatment.

### 2.3. Endpoints

1. Curative effect: the negative conversion ratio (NCR) was assessed by cervical HPV-DNA, with the efficacy divided into three grades. Negative conversion: vaginal and cervical examinations at the follow-up visit showed that all high-risk HPV subtypes were negative; effective: some positive high-risk HPV subtypes turned negative and at least one HPV subtype remained positive; ineffective: all high-risk HPV subtypes were positive. The NCR was the percentage of negative cases in the total number of cases in the group, and the overall response rate (ORR) was the percentage of the sum of negative conversion and effective cases in the total number of cases in the group.
2. Vaginal microecology: two sterile cotton swabs were used to collect vaginal secretions from the lateral wall of the patient's vagina during the return visit. One was used to detect pH, catalase, and sialidase using the dry chemical method; the other was used for vaginal microecological examination through the microscope after smear, determining the presence of microbes such as *Trichomonas vaginalis* and *Candida*, as well as microbial density and diversity. It was considered positive when the concentration of catalase was less than 2 *μ*mL/L and when the sialidase was greater than 9 units/mol.
3. Microecological restoration: vaginal microecological restoration or normal was translated in vaginal secretion pH ≤ 4.5, and the microbial density and diversity within 10–999 bacteria/oil immersion lens, with *Lactobacillus* as the dominant flora, Nugent score ≤ 3 points [12], as well as catalase and sialidase-negative. In contrast, unrecovered vaginal microecology was indicated if the vaginal secretion pH was greater than 4.5, and microbial density and diversity were 1–9 or more than 1000 bacteria/oil immersion lens, with Gram-negative *Brevibacterium*, coccus, or miscellaneous bacteria as the dominant flora, Nugent score > 3, as well as catalase and sialidase-positive.
4. Safety: we observed and counted the cases of vaginal redness and swelling, vaginal tingling, vaginal bleeding, and cervical or vaginal neoplasms in both the groups. The total incidence of adverse events (AEs) was the percentage of these events in the total number of cases in the group.

### 2.4. Statistical Processing

The data was visualized by GraphPad Prism 6 (GraphPad Software, San Diego, USA). Counting data were expressed by case number/percentage (*n* (%)), and the chi-square test was used for comparison between groups. Mean ± standard deviation (mean ± SD) was used to represent the measurement data. The methods for intergroup and intragroup (before and after treatment) comparisons of measurement data were the independent sample *t*-test and paired *t*-test, respectively. Statistically significant differences were assumed at *P* values less than 0.05.

## 3. Results

### 3.1. Baseline Data of HPV-Infected Patients

The two cohorts differed insignificantly in age, mean age, course of disease, pathological classification, HPV genotyping, residence, family history, and other baseline data (*P* > 0.05), as given in Table 1.

### 3.2. Efficacy in HPV-Infected Patients

The NCR and ORR of RG were 57.27% and 90.90%, respectively, while those of CG were 47.78% and 72.22%, respectively. The above data revealed statistically higher NCR and ORR in RG compared with CG (*P* < 0.05), as given in Table 2.

### 3.3. Vaginal Microecology in Patients with HPV Infection

Significant differences were present in catalase-positive, sialidase-positive, abnormal microbial density, and abnormal microbial diversity between RG and CG (*P* < 0.05); while the two cohorts of patients showed no statistical significance in *Trichomonas vaginalis*-positive and *Candida*-positive (*P* < 0.05), as given in Table 3.

### 3.4. Microecological Recovery of HPV-Infected Patients

The vaginal microecology recovery rate in RG was significantly higher than that in CG (90.00% vs. 65.56%), while the pH and Nugent scores of vaginal secretions were significantly lower (*P* < 0.05), as shown in Figure 1.

### 3.5. Safety of Treatment in HPV-Infected Patients

The corresponding cases of vaginal redness and swelling, vaginal tingling, vaginal bleeding, and cervix or vaginal neoplasms were 6, 4, 4, and 0 in RG, and 4, 2, 4, and 2 in CG, respectively. RG and CG presented no statistical difference in the incidence of AEs (12.73% vs. 13.33%, *P* > 0.05), as given in Table 4.

## 4. Discussion

HPV is a DNA tumor virus, which is small, double-stranded, and nonenveloped, with many subtypes [13, 14]. After infecting cervical basal epithelium, it can complete its life cycle by relying on host cell differentiation and can control the cell cycle and even cause carcinogenic lesions by building an environment that supports viral DNA amplification [15]. HPV can be sexually transmitted, which is the trigger of almost all CC lesions [16]. We found that lacidophilin vaginal capsules have beneficial effects on the curative effect and microecological restoration of HPV-infected patients and hereby report the findings in detail.

We enrolled 200 patients with HPV infection and grouped them into two groups, in which CG was treated with rh-IFN-*α*2b and RG was treated with lacidophilin vaginal capsules on the basis of CG. The results identified statistically higher NCR and ORR under the combined intervention of lacidophilin vaginal capsules plus rh-IFN-*α*2b compared with rh-IFN-*α*2b intervention alone. After being placed in the human cervix, lacidophilin vaginal capsules can induce the growth of LAB that generate lactic acid, bacteriocin, and biosurfactant to form an anti-infection barrier mucosa, so as to competitively check and balance and even inhibit the reproduction of harmful pathogenic bacteria and restore the balance of vaginal microecological flora, thus achieving the therapeutic purpose [17]. In the vaginal microecological evaluation, the incidence rates of catalase-positive, sialidase-positive, abnormal microbial density, and abnormal microbial diversity were found to be significantly lower in RG, while no significant differences were determined in *Trichomonas vaginalis*-positive and *Candida*-positive. It indicates that the vaginal microecology of patients with lacidophilin vaginal capsule intervention is generally better. Previous studies have shown that the dynamic balance mechanism of vaginal microecology can be affected by microbial diversity, density, reproduction rate, and host status, and once this balance is maladjusted, it is easy to induce microecological infectious diseases, such as trichomoniasis vaginitis and bacterial vaginosis [18, 19]. Furthermore, the vaginal microecological recovery rate of patients additionally treated with lacidophilin vaginal capsules was found to be markedly higher, with statistically lower vaginal secretion pH and Nugent scores. Previous evidence has shown that lacidophilin vaginal capsules have the function of converting monosaccharides generated by glycogen into lactose in the vaginal microecological environment, which can effectively maintain the stability of vaginal acidic environment and correct the disorder of vaginal flora [20]. In terms of safety, we mainly recorded the cases of vaginal redness and swelling, vaginal tingling, vaginal bleeding, and cervical or vaginal neoplasms in HPV-infected patients. Although there is one more drug in RG, the incidence of AEs was no different from that in CG, suggesting a higher safety profile of the treatment implemented in RG. In the research of Verdenelli et al. [21], probiotic suppositories containing LAB not only restored and maintained normal vaginal microflora but were also well tolerated and beneficial to promote women's vaginal health, which has certain similarities with the results of this study.

The main contribution of this study to the drug treatment of HPV-infected patients is to confirm the effectiveness of lacidophilin vaginal capsules in such a patient population, which can play a therapeutic role in promoting microecological recovery, inhibiting serum inflammatory factors, and reducing the incidence of grade III-IV AEs, providing a reliable basis for drug selection and prevention of CC in patients with HPV infection. There are still some limitations that need to be taken into consideration. First of all, long-term follow-up has not been carried out, which if supplemented for prognostic analysis, can help further understand the impacts of the two treatments on the prognosis of HPV-infected patients; second, conducting animal experiments for basic research can help further understand the therapeutic mechanism of lacidophilin vaginal capsules in HPV-infected patients; finally, the sample size should be increased to further improve the accuracy of experimental results.

Taken together, with certain safety, lacidophilin vaginal capsules can significantly improve the curative effect of HPV-infected patients, maintain their vaginal microecological balance, and inhibit inflammation, which is worthy of clinical promotion.

## Figures and Tables

**Figure 1:** Microecological recovery of HPV-infected patients. (a) The vaginal microecological recovery rate of patients in the two groups. (b) The pH of vaginal secretions in the two groups. (c) Nugent scores of patients in the two groups. ^*∗∗*^*P* < 0.01.

**Table 1:** Baseline data of HPV-infected patients (*n* (%), mean ± SD).

Factors	*n*	Control group (*n* = 90)	Research group (*n* = 110)	*χ * ^2^/*t*	*P* value
Age (years)				0.034	0.853
<30	103	47 (52.00)	56 (50.91)		
≥30	97	43 (47.78)	54 (49.09)		
Average age (years)	200	29.71 ± 5.68	30.76 ± 8.14	1.035	0.302
Course of the disease (years)	200	2.25 ± 1.05	2.49 ± 1.19	1.495	0.136
Pathological classification				0.459	0.498
HPV single infection	151	70 (77.78)	81 (73.64)		
LSIL	49	20 (22.22)	29 (26.36)		
HPV genotyping				0.924	0.630
HPV 16/18-positive	122	57 (63.33)	65 (59.09)		
Positive for other 12 HPV types	44	17 (18.89)	27 (24.55)		
Positive for HPV 16/18 and other 12 types	34	16 (17.78)	18 (16.36)		
Place of residence				0.825	0.364
Urban	142	61 (67.78)	81 (73.64)		
Rural	58	29 (32.22)	29 (26.36)		
Family history				1.475	0.225
None	159	75 (83.33)	84 (76.36)		
With	41	15 (16.67)	26 (23.64)		

**Table 2:** Efficacy of patients with HPV infection (*n* (%)).

Group	*n*	Negative conversion of HPV			Total effective rate (%)
		Negative conversion	Effective	Ineffective	
Control group	90	43 (47.78)	22 (24.44)	25 (27.78)	65 (72.22)
Research group	110	63 (57.27)	32 (29.09)	15 (13.64)	100 (90.90)
*χ* ^2^ value		6.187			11.973
*P* value		0.045			<0.001

**Table 3:** Vaginal microecology of HPV-infected patients (*n* (%)).

Category	Control group (*n* = 90)	Research group (*n* = 110)	*χ* ^2^ value	*P* value
Catalase-positive	11 (12.22)	3 (2.73)	6.855	0.009
Sialidase-positive	11 (12.22)	4 (3.64)	5.260	0.022
*Trichomonas vaginalis*-positive	10 (11.11)	5 (4.55)	3.076	0.080
*Candida*-positive	7 (7.78)	3 (2.73)	2.658	0.103
Abnormal microbial density	20 (22.22)	7 (6.36)	10.661	0.001
Abnormal microbial diversity	15 (16.67)	6 (5.45)	6.622	0.010

**Table 4:** Safety analysis of patients with HPV infection (*n* (%)).

Category	Control group (*n* = 90)	Research group (*n* = 110)	*χ* ^2^ value	*P* value
Vaginal redness and swelling	4 (4.44)	6 (5.45)	—	—
Vaginal tingling	2 (2.22)	4 (3.64)	—	—
Vaginal bleeding	4 (4.44)	4 (3.64)	—	—
Cervical or vaginal neoplasms	2 (2.22)	0 (0.00)	—	—
Total	12 (13.33)	14 (12.73)	0.016	0.899

## Data Availability

The data used to support the findings of this study are available from the corresponding author upon request.
